The article "Association between Elderly Sarcopenia and Inflammatory Cytokine Interleukin-17: A Cross-Sectional Study" was retracted in 2023. Reasons: signs of a paper mill; suspected computer-generated content; unreliable results or conclusions; concerns about the data.

# Association between Elderly Sarcopenia and Inflammatory Cytokine Interleukin-17: A Cross-Sectional Study

**DOI:** 10.1155/2023/4839210

**Published:** 2023-02-22

**Authors:** Lu Xiong, Ying Chen, Xiao Dong, Yunqian Li, Min Zeng, Kai Liu

**Affiliations:** ^1^Geriatric Center, Hainan General Hospital (Hainan Affiliated Hospital of Hainan Medical University), Haikou, Hainan 570311, China; ^2^Medical Laboratory Center, Hainan General Hospital (Hainan Affiliated Hospital of Hainan Medical University), Haikou, Hainan 570311, China

## Abstract

Aging slows down the mechanisms behind skeletal muscle weakening and mobility. Increases in inflammation brought on by aging may contribute to some characteristics of sarcopenia. As a result of population aging worldwide, sarcopenia, an age-related disease, has become a huge burden on both individuals and society as a whole. The study of the morbidity mechanism and available sarcopenia treatments has received more attention. The inflammatory response may be one of the most important methods behind the pathophysiology of sarcopenia in the aged, according to the background of the study. This anti-inflammatory cytokine inhibits the ability of human monocytes and macrophages to induce inflammation as well as the production of cytokines like IL-6. Here, we investigate the association between sarcopenia and interleukin-17 (IL-17), an inflammatory cytokine in the aged. There were 262 subjects aged 61-90 years who were screened for sarcopenia in Hainan General Hospital. The subjects were divided into 45 males and 60 females aged 65-79 years (average age: 72.00 ± 4.31 years). 105 patients without sarcopenia were randomly selected among 157 participants. It included 50 males and 55 females, aged 61-76 years (mean age: 69.10 ± 4.55 years) as per the standard definition of the Asian Working Group for Sarcopenia (AWGS). The “skeletal muscle index” (SMI), “hand grip strength” (HGS), “gait speed” (GS), “biochemical indexes,” “serum IL-17 level,” nutritional status, and past medical history of the two groups were evaluated and compared. Compared with the participants without sarcopenia, sarcopenia patients had higher average age; less physical exercise; lower total scores of BMI, pre-ALB, IL-17, and SPPB; and a higher proportion of malnutrition risk (all *P* < 0.05). By “ROC curve analysis,” the best critical point was IL-17 in the growth of sarcopenia. The area that comes under ROC (AUROC) value was 0.627 (95% CI = 0.552, 0.702, *P* = 0.002). The ideal threshold value for IL-17 to estimate sarcopenia was 18.5 pg/mL. In the unadjusted model, IL-17 was considerably linked to sarcopenia (OR = 1.123, 95% CI = 1.037-1.215, *P* = 0.004). After the covariate adjustment observed in the complete adjustment model (OR = 1.111, 95% CI = 1.004-1.229, *P* = 0.002), this significance still exists. The results of this study suggest a strong relationship between sarcopenia and IL-17. This study will look at IL-17's potential to serve as a key sarcopenia indicator. This trial is registered with ChiCTR2200022590.

The article "Association between Elderly Sarcopenia and Inflammatory Cytokine Interleukin-17: A Cross-Sectional Study" was retracted in 2023. Reasons: signs of a paper mill; suspected computer-generated content; unreliable results or conclusions; concerns about the data.

## 1. Introduction

Population aging has emerged as a top concern of many nations; it is simple and easy to overlook age-related sarcopenia. An indication of aging is chronic inflammation. Sarcopenia is now a frequent condition among the elderly, placing a significant burden on the global healthcare system and society [1]. Age-related muscle loss was originally used to represent sarcopenia [2]. The immune system is expected to remodel as we age due in large part to cytokine dysregulation, and the failure to accurately control systemic inflammation is thought to be a symptom of unsuccessful aging. When cytokine expression patterns alter and tend to become more proinflammatory over time, it has been labeled “inflammaging.” The current definition, however, covers chronic disease-related muscle loss, physical inactivity or impaired activity, and undernourishment [3]. Immune cells are redirected to infected or injured tissues during inflammation. The development of autoimmune, allergy, and cancerous disorders is heavily influenced by chronic inflammation. Due to its role in autoimmune illnesses in both humans and mice, interleukin-17 (IL-17) is the founding member of a new cytokine family that has lately garnered popularity. Sarcopenia can increase the rate of falls [4] leading to fractures [4] and increased risk of disability [5] and loss of self-care ability in the elderly. Timely and early recognition and treatment of sarcopenia and a better understanding of the adverse outcomes of sarcopenia are conducive to maintaining the health and better life quality of aged people. By using the AWGS 2014 criteria, the analysis of epidemiology studies from Asian countries finds out that there is a 5.5% to 25.7% occurrence of sarcopenia with male predominance. There is a high prevalence of 5.1%-21.0% in men in comparison to 4.1%-16.3% in women [6]. The loss in muscle glycolysis ability that comes with aging is facilitated by the NLRP3 inflammasome. Age-related alterations in muscle glycolytic enzyme activity and myofiber size are decreased when NLRP3 is eliminated. The proinflammatory cytokine IL-6, the anti-inflammatory cytokine IL-10, and the IL-6/IL-10 ratios were all found to be increased in senior sarcopenia patients. Sarcopenia was associated with elevated levels of the proinflammatory cytokine IL-6, the anti-inflammatory cytokine IL-10, and IL-6/IL-10 ratios. By increasing autophagy activity to hasten the clearance of immunological mediators, the NOD-like receptor 3 (NLRP3) inflammasome normally fine-tunes the course of the innate immune response it has triggered. The autophagy response is reduced as we age and develop age-related disorders, immunological mediators are still active, and inflammation is prolonged.

The article "Association between Elderly Sarcopenia and Inflammatory Cytokine Interleukin-17: A Cross-Sectional Study" was retracted in 2023. Reasons: signs of a paper mill; suspected computer-generated content; unreliable results or conclusions; concerns about the data.

The causes of sarcopenia may be multifaceted including muscle loss [7], endocrine changes [8], chronic diseases [9], chronic inflammation [10], insulin resistance [11], and nutritional deficiencies [12]. Although there are many factors related to the pathophysiology of sarcopenia, its pathophysiological mechanism is still difficult to determine. The inflammatory response is an important pathological process for the body to resist harmful factors in vivo and in vitro, which often plays a positive role in protecting the body. However, too long-lasting inflammatory response often leads to many chronic diseases (such as type 2 diabetes and osteoporosis) and other age-associated diseases (such as muscle atrophy, weakness, and even death) [13]. Numerous studies [14–16] have demonstrated a relationship between sarcopenia and chronic inflammation. As a result of the activation of inflammatory cells like mononuclear macrophages, which releases inflammatory mediators including tumor necrosis factor (TNF) and interleukin-1 (IL-1), the body's defense response is also aided by numerous inflammatory factors in chronic inflammation [17].

IL-17 and IL-17F form biologically active heterodimers with moderate potency for inducing inflammatory genes when compared to homodimers. Interleukin-17 (IL-17A, generally known as IL-17) is one of the cytokines that was cloned in 1993, but it remained unclear throughout the 1990s and early 2000s. Several early investigations suggested that this cytokine was raised in human inflammatory or autoimmune illnesses and was expressed in a noncanonical T helper cell population [18]. The study reported that the rate of circulating proinflammatory cytokines (such as IL-6 and TNF-*α*) was raised in aged patients with sarcopenia [19]. Uncertainty surrounds the function of anti-inflammatory cytokines in sarcopenic elderly people. It is well recognized that no research has been done to determine whether IL-17 may have a role in sarcopenia patients. To research this issue, we determined the link between IL-17 levels and sarcopenia in elderly patients and measured the blood concentration of inflammatory cytokines.

## 2. Methods and Material

### 2.1. Research Objects

At the Geriatrics Center of Hainan General Hospital in China, between May 2019 and May 2020, a total of 262 elderly people aged between 61 and 90 were assessed as sarcopenia. In line with AWGS [6], sarcopenia was identified in 105 individuals. All participants had to be older than 60 and be able to stand and move around on their own. The analysis is based on criteria 1 (low muscle mass) plus criteria 2 (low muscle strength) or criteria 3 (poor physical performance), suggested amputation of the skeletal muscle mass measurements in the extremities point values (28 kg for men and 18 kg for women), and normal gait speed (1 m/s), as per the AWGS criteria for sarcopenia in the elderly [6].

The article "Association between Elderly Sarcopenia and Inflammatory Cytokine Interleukin-17: A Cross-Sectional Study" was retracted in 2023. Reasons: signs of a paper mill; suspected computer-generated content; unreliable results or conclusions; concerns about the data.

#### 2.1.1. Exclusion Criteria

The experimental subjects are those who are under the age of 60; have tumors that are obviously malignant; are bedridden due to severe stroke, heart failure, renal problems, fractures, and other diseases; are subject to severe endocrine diseases and poor management; and have infectious diseases, autoimmune diseases, and a history of mental illness.  Figure 1 shows the study's flowchart. We included 60 women and 45 males between the ages of 65 and 79 (mean age: 72.00 ± 4.31 years). 50 men and 55 women between the ages of 61 and 76 were chosen at random from 157 volunteers to make up the 105 patients without sarcopenia (mean age: 69.10 ± 4.55 years).

### 2.2. Sarcopenia Measurement

According to the AWGS [6] definition, sarcopenia is characterized by decreased muscular mass, low muscle strength, or/and low physical performance. Using DXA, muscle mass was evaluated (Medix DR, Medilink, France). An experienced technician performed all the scans. The mass of the skeletal muscles in the arm and leg was added to determine the appendiceal skeletal muscle (ASM; kg). ASM subject to division by the square of height (m^2^) yields the skeletal muscle index (SMI) [6]. Male SMI (7 kg/m^2^) and female SMI (5.4 kg/m^2^) were used to identify low muscle mass [6].

Using a Xiangshan electronic grip tester, grip strength (HGS), the measure of muscle strength was determined (Zhejiang, China). Three times with each hand, the subjects were instructed to use their best effort. Sarcopenia is diagnosed using the maximum HGS. The AWGS consensus standard defines low HGS as males of 28 kg and females of 18 kg [6].

During the 6-meter process, gait speed (m/s) is employed as a gauge of physical performance. Subjects of the experiment were told to walk six meters at their normal pace [6]. The results of two timed tests were compared, and sarcopenia was determined by the better test result and performance. According to the AWGS consensus cutoff point, low gait speed is defined as a gait speed of less than 1 m/s [6].

### 2.3. Life Pattern and Social Demographic Factors

- Definition criteria for regular exercise: exercised more than thrice a week, more than 30 minutes each time, and during the past 6 months at least. All of these are considered normal as regular exercises
- Smoking definition criteria: the World Health Organization defines “continuous or cumulative smoking for 6 months or more in a lifetime” as a smoker. These participants were partitioned into two groups: smokers and nonsmokers
- Definition standard of drinking: according to drinking habits, these participants were separated into two categories: drinkers and nondrinkers

The article "Association between Elderly Sarcopenia and Inflammatory Cytokine Interleukin-17: A Cross-Sectional Study" was retracted in 2023. Reasons: signs of a paper mill; suspected computer-generated content; unreliable results or conclusions; concerns about the data.

### 2.4. Laboratory Metrics

After fasting for at least 6 hours in the morning, 5 mL of cubital venous blood was drawn from each subject. Hemoglobin (Hb) and blood biochemical indicators were calculated soon after blood was drawn. The leftover serum was stored at -80°C for consequent and later testing of IL-17 levels.

### 2.5. Nutritional Risk

Using a brief form of the mini nutritional assessment, we assessed the nutritional risk (MNA-SF). Participants were deemed to be at risk of undernourishment if their scores were less than or equal to 11.

### 2.6. Quantification of IL-17 Levels

IL-17 was quantified by flow cytometry (BD FACSAria III flow cytometry, USA) and reagents from Jiangxi Saiji Biotechnology Co., Ltd. according to the requirements of reagent manufacturers with a normal reference interval of 0–20.6 pg/mL.

### 2.7. Statistical Analysis

SPSS is used for the statistical analysis of this study (version 26.0 for Windows, SPSS, Inc., Chicago, IL, USA). Indicators for continuous data were the median and interquartile range (IQR). Utilizing frequency counts and percentages, categorical data were recorded. The chi-square test and independent sample *t*-test are used, respectively, for categorical and continuous variables. To assess the strength of the connection between IL-17 and sarcopenia, odds ratios (ORs) were created using logistic regression. The strength of the relationship between IL-17 levels and grip strength, SMI, and speed was further examined in the current study using Pearson's correlation coefficients. A multivariate linear regression model with a progressively changed architecture was used to explain the connection between IL-17 and the sarcopenia component. The current study further examined the strength of the relationship between IL-17 levels and grip strength, SMI, and pace using Pearson's correlation coefficients. IL-17 and the sarcopenia components were related, and we used a multivariate linear regression model with a gradually changed design to explain this link. By using the following extended model linear regression, covariate adjustment was examined. The best IL-17 cutoff value for sarcopenia prediction was investigated using receiver operating characteristic (ROC) curve analysis.

The article "Association between Elderly Sarcopenia and Inflammatory Cytokine Interleukin-17: A Cross-Sectional Study" was retracted in 2023. Reasons: signs of a paper mill; suspected computer-generated content; unreliable results or conclusions; concerns about the data.

## 3. Results

### 3.1. Study Sample Characteristics

Table 1 shows the demographic sample. In comparison to participants without sarcopenia, sarcopenia patients had higher average age; less physical exercise; lower total scores of BMI, pre-ALB, IL-17 A, and SPPB; and a higher proportion of malnutrition risk (all *P* < 0.05).

In comparison to the no sarcopenia group, the grip strength, SMI, and walking speed in the sarcopenia group were lower and the three continuous variables were statistically significant (*P* < 0.001).

### 3.2. IL-17 and Its Association with Sarcopenia

In Table 2, we analyzed the connection between IL-17 and sarcopenia by logistic regression. In model 1, IL-17 was notably linked to sarcopenia (OR = 1.123, 95% CI = 1.037-1.215, *P* = 0.004). After the covariate adjustment observed in model 2 (OR = 1.130, 95% CI = 1.038-1.230, *P* = 0.005) and model 3 (OR = 1.111, 95% CI = 1.004-1.229, *P* = 0.002), aboriginality persisted.

By “ROC curve analysis,” Figure 2 emphasizes the best critical point of IL-17 in the growth of sarcopenia. The area that comes under ROC (AUROC) value was 0.627 (95% CI = 0.552, 0.702, *P* = 0.002). The “optimal cutoff value of 18.5 pg/mL” was established by the maximum “Youden's index” with a sensitivity of 0.829 and specificity of 0.381.

### 3.3. Association between Muscle Quality Index and IL-17

Figure 3 shows that the correlation coefficients between IL-17 and SMI, grip strength, and stride speed are -0.263, -0.202, and -0.174, respectively. The multivariate-adjusted linear analysis of the relationship between IL-17 and muscle mass index is represented in Table 3. The relationship between IL-17 and SMI (*β* = −0.263, 95% CI = −0.101, -0.034, *P* < 0.001), HGS (*β* = −0.174, 95% CI = −0.511, -0.065, *P* = 0.012), and gait speed (*β* = −0.202, 95% CI = −0.025, *P* = 0.003), showed statistical implication and importance in the unadjusted model. Similar trends were noticed in the fully adjusted model. The *β* coefficients of SMI, HGS, and gait speed were -0.212 (95% CI = −0.064, -0.015, *P* = 0.001), -0.130 (95% CI = −0.428, -0.002, *P* = 0.048), and -0.169 (95% CI = −0.022, -0.003, *P* = 0.011).

## 4. Discussion

This study examines the relationship between IL-17 levels and the type of sarcopenia in representative samples of older sarcopenic patients. Our findings demonstrated a strong correlation between IL-17 levels and sarcopenia. As we know, the role of serum IL-17 in predicting sarcopenia was investigated for the first time in this study. Additionally, the NLRP3 inflammasome plays a role in the reduction in muscle glycolysis that comes with age. Age-related alterations in muscle glycolytic enzyme activity and myofiber size are decreased when NLRP3 is eliminated.

The article "Association between Elderly Sarcopenia and Inflammatory Cytokine Interleukin-17: A Cross-Sectional Study" was retracted in 2023. Reasons: signs of a paper mill; suspected computer-generated content; unreliable results or conclusions; concerns about the data.

Studies have stressed the connection between (chronic) systemic inflammation and a decline in skeletal muscle function [20], as well as aging, which is accompanied by older people's greater inflammatory activity levels [21]. Some scholars have observed that in elderly patients with sarcopenia, the levels of circulating proinflammatory markers IL-6 [22], IL-10 [22], and TNF-*α* [23] went up. Sarcopenia is characterized by reduced muscle mass, weakened muscle strength, and poor physical performance and is caused by the production of inflammatory cytokines by skeletal muscle cells and inflammatory cells. It makes bad outcomes more likely to occur [24]. The rise in IL-17 levels that we saw in sarcopenia patients was confirmed by some studies. IL-17 impairs muscular contraction and weakens skeletal muscle [25]. ER stress, calcium imbalance, and the release of IL-6 and CC-chemokine ligand 20 are all stimulated in skeletal muscle by IL-17 alone (or in conjunction with TNF- or IL-1) (CCL20). All of these factors encourage inflammatory immune cell infiltration, and IL-17 is linked to the suppression of myogenic differentiation and muscle cell migration [25].

The aged patients will have chronic low-grade inflammation when getting old [26]. Aging is the decline of the overall body systems, organs, and tissues, which is related to the decrease in adaptability and intrinsic immunity. This is also called immune aging which exhibits an increase of proinflammatory cytokines in the blood without obvious induction [27]. Research on the direct outcome of IL-17 on muscle cells is restricted. Most of the research is conducted in the context of myocarditis. IL-17 has a proinflammatory impact on human myoblasts by raising the secretion of IL-6. However, IL-6 can regulate carbohydrate and lipid metabolism, promote the rise and proliferation of muscle satellite cells, or lead to muscle atrophy [25]. In addition, the growth hormone-insulin-like growth factor-I axis is the key medium for skeletal muscle growth and adaptation [25]. Autocrine/paracrine IGF-I is proven to adjust the compensatory adaptation of skeletal muscle and muscle growth. In addition, excessive expression of IL-6 will interfere with GH-IGF-I axis, leading to skeletal muscle atrophy [25]. Cytokine dysregulation is expected to play a crucial part in the remodeling of the immune system as we age, with studies showing a failure to precisely modulate systemic inflammation, which appears to be a marker of unsuccessful aging. This change in cytokine production pattern with a steady tendency toward a proinflammatory phenotype is known as “inflame-aging” [28].

The article "Association between Elderly Sarcopenia and Inflammatory Cytokine Interleukin-17: A Cross-Sectional Study" was retracted in 2023. Reasons: signs of a paper mill; suspected computer-generated content; unreliable results or conclusions; concerns about the data.

In older individuals with sarcopenia, the study showed that IL-17 was inversely correlated with grip strength and walking speed. Walking speed and grip strength are indicators of physical function in the elderly. At present, there is no separate research report on IL-17 and walking speed, but Kositsawat et al. [29] found that after managing other biomarkers and potential confounding factors, IL-6 became the only biomarker independent of walking speed. Chen et al. [30] discovered that low muscle strength and low-speed gait have a negative link with IL-12. Both are inflammatory factors. In our study, a multiple linear regression model was used to adjust, and finally, it was found that for every unit increase in IL-17, grip strength decreased by 13% and walking speed decreased by 16.9%. Inflammasome activity, cytokine production, antigen presentation, and lymphocyte function are all impacted by the dysregulation of autophagy, which has significant consequences on the innate immune response, aging, and age-related illnesses. A most significant characteristic of sarcopenia in aged patients is the decrease in grip strength. A study in the hemodialysis population found that low grip strength is related to poor functional ability and high inflammation [31]. At present, there is no report on the correlation between IL-17 and grip strength, but a meta-analysis result also shows that plasma IL-6 is negatively correlated with grip strength [32]. The impact of IL-17 is proinflammatory on human myoblasts as it increases the discharge of IL-6. According to [33], the older mice's skeletal muscles have increased activity of the inflammatory caspase-1. The NLRP3/caspase-1 inflammasome plays a role in mice's age-related loss of muscle mass and function (relative to body mass). They could not discover any proof of changes in systemic inflammatory indicators brought on by NLRP3 throughout aging. Instead, they discovered that the deletion of NLRP3 diminished muscle-intrinsic reactions associated with glycolytic metabolism. The proteolysis/inactivation of GAPDH, a rate-limiting enzyme in glycolysis, and the age-related reduction in the size of glycolytic myofibers were both dependent on NLRP3.

This study was the first to investigate how serum IL-17 affected the likelihood of developing sarcopenia. The results suggested a substantial association between IL-17 and sarcopenia in both men and women. The level of serum IL-17 may be a useful signal to assess the threat of sarcopenia in a clinical setting, even though additional research and investigations are needed to confirm the potential mechanism.

The article "Association between Elderly Sarcopenia and Inflammatory Cytokine Interleukin-17: A Cross-Sectional Study" was retracted in 2023. Reasons: signs of a paper mill; suspected computer-generated content; unreliable results or conclusions; concerns about the data.

## 5. Conclusion

Age-related decline in muscle glycolytic capacity is facilitated by the NLRP3 inflammasome. The reduction in the number of glycolytic myofibers and the decreased activity of glycolytic enzymes in muscle with aging are both lessened by the deletion of NLRP3. This study examines the relationship between IL-17 levels and the type of sarcopenia in representative samples of older sarcopenic patients. Our findings demonstrated a strong correlation between IL-17 levels and sarcopenia. The loss in muscle glycolysis ability that comes with aging is facilitated by the NLRP3 inflammasome. Age-related alterations in muscle glycolytic enzyme activity and myofiber size are decreased when NLRP3 is eliminated. The proinflammatory cytokine IL-6, the anti-inflammatory cytokine IL-10, and the IL-6/IL-10 ratios were all found to be increased in senior sarcopenia patients. Sarcopenia was associated with elevated levels of the proinflammatory cytokine IL-6, the anti-inflammatory cytokine IL-10, and IL-6/IL-10 ratios. By increasing autophagy activity to hasten the clearance of immunological mediators, the NOD-like receptor 3 (NLRP3) inflammasome normally fine-tunes the course of the innate immune response it has triggered. The autophagy response is reduced as we age and develop age-related disorders, immunological mediators are still active, and inflammation is prolonged. Additionally, the selection bias in the current study design may result in an incorrect expression of the connection. The patients' cognitive condition, drug use, and dietary health are crucial aspects of sarcopenia, but they are completely ignored. Therefore, the influence of confusion bias cannot be ignored.

## Figures and Tables

**Figure 1:** Flow chart representation of the analysis steps performed in the study.

**Figure 2:** Receiver operating characteristic curve analysis.

**Figure 3:** Pearson's correlation coefficient between IL-17 and muscle quality index.

**Table 1:** Basic characteristics of study sample.

Variable	Sarcopenia (*n* = 105)	Nonsarcopenia (*n* = 105)	*P*
Age (y)	72.00 ± 4.31	69.10 ± 4.55	<0.001
Male (%)	45 (42.86)	50 (47.62)	0.488
BMI (kg/m^2^)	23.91 ± 2.63	24.91 ± 2.85	0.009
Hypertension (%)	45 (42.86)	47 (44.76)	0.781
Diabetes (%)	24 (22.86)	26 (24.76)	0.746
Coronary artery disease (%)	25 (23.81)	24 (22.86)	0.870
Smoke (%)	31 (29.52)	29 (27.62)	0.760
Drink (%)	28 (26.67)	30 (28.57)	0.758
Sport (%)	10 (9.52)	23 (21.90)	0.014
SMI (kg/m^2^)	5.51 ± 0.53	6.91 ± 0.64	<0.001
Grip strength (kg)	19.85 ± 4.10	27.16 ± 5.05	<0.001
Gait speed (m/s)	0.84 ± 0.21	1.15 ± 0.22	<0.001
MNA-SF ≤ 11 (%)	78 (74.29)	59 (56.19)	0.006
TG (mmol/L)	1.46 ± 0.29	1.48 ± 0.28	0.746
TCHOL (mmol/L)	2.50 ± 0.54	2.54 ± 0.49	0.649
LDL-C (mmol/L)	3.01 ± 0.54	3.08 ± 0.51	0.375
Hb (g/L)	124.42 ± 13.68	125.52 ± 14.64	0.573
ALB (g/L)	36.84 ± 6.99	38.67 ± 7.19	0.063
Pre-ALB (mg/L)	252.07 ± 49.90	300.58 ± 44.22	<0.001

The article "Association between Elderly Sarcopenia and Inflammatory Cytokine Interleukin-17: A Cross-Sectional Study" was retracted in 2023. Reasons: signs of a paper mill; suspected computer-generated content; unreliable results or conclusions; concerns about the data.

**Table 2:** The logistic regression results of IL-17 in predicting sarcopenia.

		Model 1	Model 2	Model 3
Sarcopenia	Odds ratio (95% CI)	1.123 (1.037-1.215)	1.130 (1.038-1.230)	1.111 (1.004-1.229)
	*P* value	0.004	0.005	0.041

Model 1: unadjusted; model 2: adjusted for age and BMI; model 3: model 2 + prealbumin, hemoglobin, MNA-SF, and SPPB.

**Table 3:** Association between IL-17 and muscle quality index.

	SMI		Grip strength		Gait speed	
	*β*(95% CI)	*P*	*β*(95% CI)	*P*	*β*(95% CI)	*P*
Model 1	-0.263 (-0.101, -0.034)	<0.001	-0.174 (-0.511, -0.065)	0.012	-0.202 (-0.025, 0.005)	0.003
Model 2	-0.252 (-0.097, -0.032)	<0.001	-0.164 (-0.490, -0.056)	0.014	-0.193 (-0.024, -0.005)	0.004
Model 3	-0.212 (-0.064, -0.015)	0.001	-0.130 (-0.428, -0.002)	0.048	-0.169 (-0.022, -0.003)	0.011

Model 1: unadjusted; model 2: adjusted for age and BMI; model 3: model 2 + prealbumin, hemoglobin, MNA-SF, and SPPB.

## Data Availability

The datasets used in this paper are available from the corresponding author upon request.
